# Research on Video Quality Evaluation of Sparring Motion Based on BPNN Perception

**DOI:** 10.1155/2021/9615290

**Published:** 2021-12-27

**Authors:** Zhao Changbi, Wang Jinjuan, Ke Li

**Affiliations:** ^1^Department of Physical Education, Dalian University of Foreign Languages, Dalian, Liaoning 116044, China; ^2^School of Physical Education, Liaoning Normal University, Dalian, Liaoning 116029, China; ^3^Institute of Physical Education, Huazhong University of Science and Technology, Wuhan, Hubei 430074, China; ^4^School of Physical Education and Sports Science, Jishou University, Jishou 416000, China

## Abstract

The quality of boxing video is affected by many factors. For example, it needs to be compressed and encoded before transmission. In the process of transmission, it will encounter network conditions such as packet loss and jitter, which will affect the video quality. Combined with the proposed nine characteristic parameters affecting video quality, this paper proposes an architecture of video quality evaluation system. Aiming at the compression damage and transmission damage of leisure sports video, a video quality evaluation algorithm based on BP neural network (BPNN) is proposed. A specific Wushu video quality evaluation algorithm system is implemented. The system takes the result of feature engineering of 9 feature parameters of boxing video as the input and the subjective quality score of video as the training output. The mapping relationship is established by BPNN algorithm, and the objective evaluation quality of boxing video is finally obtained. The results show that using the neural network analysis model, the characteristic parameters of compression damage and transmission damage used in this paper can get better evaluation results. Compared with the comparison algorithm, the accuracy of the video quality evaluation method proposed in this paper has been greatly improved. The subjective characteristics of users are evaluated quantitatively and added to the objective video quality evaluation model in this paper, so as to make the video evaluation more accurate and closer to users.

## 1. Introduction

With the booming development of communication technology in the information age, the network has become an essential part of society. Sparring sports information can be transmitted in the network in various forms such as voice, image, and video. And, in today's era, with more and more information and better network services, it is natural that casual sports video information plays a more important role and video services have become an important business for network service providers because casual sports videos carry more information and the presentation form that people are more willing to accept [1–4].

The video of casual sports is played in real time in streaming form through network transmission. Since the video is played in streaming form, users do not need to wait until the whole video is downloaded and can play it while downloading. Nowadays, the video service is a very important part of the process of receiving information about sparring sports for sparring athletes and fans and has become an indispensable part of the life of sparring sports fans [5, 6]. For example, the video service of sparring sports includes sparring movies on demand and live broadcast of sparring matches. In the past, the traditional video of sparring sports was played directly without network transmission, and some information was lost and distorted when the video was compressed. Compared with the video transmitted without network, the quality of the network transmission of the casual sports video will receive damage not only during compression but also during transmission. In the transmission network of video, packet loss, delay, jitter, and other problems will affect the quality of video, causing blurred images and stagnant playback of casual sports video, making the user viewing experience degraded. And, in order to improve the quality of casual sports video, it is firstly needed to effectively evaluate and quantify the quality of casual sports video, so the quality assessment of casual sports video has become more and more important [7].

As people's interest in sports, especially sparring, increases, sparring video quality has become a key concern for users, including the following two points: first, the quality of sparring video images is required; just SD quality video can no longer meet the needs of users; HD, ultra HD, and even Blu-ray quality sparring videos are increasingly appearing in today's video services; second, the smoothness of sparring video playback, for any real-time online video service and frequent and long playback lags seriously affects the users' experience. So, ensuring video clarity while enabling smooth playback of casual sports videos is also a key concern for users. Therefore, how to effectively evaluate the quality of casual sports videos to provide a basis for improving the quality of casual sports video services and user experience is of great practical significance [8].

Aiming at the compression damage and transmission damage of leisure sports video, this paper creatively proposes a video quality evaluation algorithm based on BP neural network (BPNN). A specific Wushu video quality evaluation algorithm system is implemented. The system takes the feature engineering results of 9 feature parameters of boxing video as the input and the subjective quality score of video as the training output. The mapping relationship is established through BPNN algorithm, and finally the objective evaluation of boxing video quality is obtained. In this paper, the subjective characteristics of users are quantitatively evaluated and added to the objective video quality evaluation model to make the video evaluation more accurate and closer to users.

The structure of this paper is mainly arranged as follows: Chapter 1 introduces the research background, significance, and structure of this paper on video quality evaluation of sparring sports. Chapter 2 introduces the related research on video quality evaluation in recent years and the main research content of this paper. Chapter 3 analyzes the damage suffered by the sparring sports video during compression and transmission, extracts the feature parameters for evaluating the quality of sparring sports video based on the damage analysis, and analyzes the correlation between these feature parameters and the quality score. Chapter 4 proposes a BPNN-based quality evaluation algorithm model for sparring sports video, discusses the specific implementation method of the model, and deploys the implementation in practice. Chapter 5 introduces the evaluation criteria of the quality evaluation algorithm and verifies the superiority of the algorithm using experimental simulations. Chapter 6 summarizes the full text and summarizes the results of this paper, while proposing the shortcomings of this paper and the research directions for the next work.

## 2. The Related Works

Since the last few years, studies on the quality evaluation of casual sports videos disseminated through the Internet have received increasing attention, and many institutions and laboratories have been involved in related studies [9, 10]. There are many laboratories in universities that study video quality, such as the LIVE Lab at the University of Texas, which provides many video quality-related datasets. Video quality evaluation methods can usually be divided into two main categories: subjective quality evaluation methods and objective quality evaluation methods [11–13]. For subjective quality evaluation methods, it is necessary to first find a group of test users who meet the requirements and then let these users watch the same multiple video sequences and quantify the subjective quality evaluation results based on the feedback from these users. This type of method requires that the number of users should not be too small and also requires a very strict testing environment; otherwise the evaluation results will be highly contingent and volatile [14]. In contrast, objective quality evaluation algorithms are more feasible because they use computers to automatically evaluate video quality without the need for test users. The objective quality evaluation algorithm aims to calculate a video quality score that matches the subjective evaluation result, and it is usually considered that the closer the objective quality evaluation result is to the subjective quality evaluation result, the more accurate the objective quality evaluation algorithm is [15–19].

Video quality evaluation of casual sports has received much attention and has been rapidly developed in recent years [20, 21]. The current research on video quality evaluation methods focuses on the following two aspects. (1) Real-time objective unreferenced video quality evaluation research: for many online video applications, real-time quality evaluation is of practical value. Meanwhile, for network applications, it is certainly unrealistic to obtain the original video source before compressed transmission or to evaluate the video quality by user groups, so objective reference-free quality evaluation algorithms are undoubtedly the focus of the moment [22–24]. (2) Video impact factor research: there are very many factors affecting video quality, and reference to all factors to evaluate video quality is unrealistic from the point of view of implementation difficulty and time complexity [25]. So, usually the main influencing factors of video quality are extracted and from that the video quality is evaluated. Then, which factors are extracted, how to extract and calculate each factor, and how to derive the final video quality score from each influencing factor are the main research points of each video quality assessment method [26].

Although there are many methods for video quality evaluation, there is no uniform standard yet. So, video quality evaluation is still an important issue. In addition, the current research has achieved some results, which can meet the demand for the quality of casual sports video in daily life. However, because there are more degradation factors causing the video quality and the video needs to consider the feature information in the time domain, it is much more difficult compared with the picture quality evaluation. Therefore, the performance of the current algorithm is not particularly good, and researchers still have a long way to go in this area. This paper makes a study of the video quality evaluation of sparring sports, taking into account today's trends. In this paper, the following results are proposed for the video quality evaluation of sparring sports: the video quality impairment of sparring sports is studied, and compression impairment and transmission impairment are analyzed. Three feature parameters, namely, quantization parameter, ambiguity degree, and the number of jump macroblocks, are proposed for compression impairment, and six feature parameters, namely, strain degree, block effect degree, aggregation block effect degree, initial buffering delay, average duration of jamming, and jamming frequency, are proposed for transmission impairment, and the correlation between each of the proposed feature parameters and the quality of scattered sports video is also analyzed. A model for evaluating the quality of scattering sports video is established. The feature parameters are extracted from the sparring sports video and the BPNN network model is used to evaluate the video quality. Meanwhile, the concrete implementation of this scattering sports video quality evaluation model is given from a practical point of view, and each specific process of the system implementation is given, and finally the superiority of the model is demonstrated by comparing the algorithm with other scattering sports video quality evaluation methods.

## 3. Sporadic Video Quality Feature Extraction

### 3.1. Compression Damage Characteristic Parameters Selection

In video quality evaluation, compression impairment is a factor that must be considered, and the degree of compression impairment can greatly affect the video source quality. In this section, two coding parameters, quantization parameter and number of jump macroblocks, are extracted as features, as well as the evaluation of fuzzy distortion to obtain the fuzziness as a feature parameter, while evaluating the video compression quality impairment.

#### 3.1.1. Quantization Parameter (QP)

The distortion of the video in the compression process mainly lies in the quantization step, and the quantization parameter is an important parameter to determine the degree of quantization. The smaller the quantization parameter, the smaller the quantization step (QStep), and the larger the amount of compressed video data, but at the same time the smaller the degree of distortion after decoding, while if the quantization parameter is larger, there will be a larger quantization step. For a frame, there are three components of YUV, which are quantized separately with different quantization parameters and value ranges. For the coding of luminance component, there are 52 quantization steps, so the quantization parameters are from 0 to 51; for the coding of chrominance component, there are 40 quantization steps, and the quantization parameters are from 0 to 39.

#### 3.1.2. Blurriness

The blurriness of the video is often an important factor affecting the video quality, and this can be caused by a variety of reasons, such as intraframe prediction and motion compensation for interframe prediction. Therefore, in this paper, the blurriness is extracted as another feature to evaluate the video quality. In this paper, we use the method of measuring the blurring degree of a video by the loss of video details after filtering the video. First, this paper uses a Gaussian filter to filter the video. The Gaussian filtering process is as follows.

(1) $$\begin{array}{c} I^{\prime }\left(x,y\right)=I\left(x,y\right)\cdot G, \end{array}$$

where *I*′(*x*, *y*) is the filtered image point information and is a *G*5 × 5 Gaussian filter matrix:

(2) $$\begin{array}{c} G=\frac{1}{273}\left[\begin{array}{ccccc} 1 & 4 & 7 & 4 & 1\\ 4 & 16 & 26 & 16 & 4\\ 7 & 26 & 41 & 26 & 7\\ 4 & 16 & 26 & 16 & 4\\ 1 & 4 & 7 & 4 & 1 \end{array}\right]. \end{array}$$

Ultimately, the blurriness of a frame is defined as follows, where *w* and *h* are the width and height of a frame, respectively:

(3) $$\begin{array}{c} D_{\text{Blur}}=\frac{\sum_{x<w,y<h}\left|I\left(x,y\right)-I^{\prime }\left(x,y\right)\right|}{w\times h}. \end{array}$$

#### 3.1.3. Number of Jump Macroblocks

When H.264 is encoded, interframe prediction and intraframe prediction are performed. For macroblocks within the flat region of nonkey frames, they are often defined as jump macroblocks. In order to improve the coding efficiency, jump macroblocks are encoded without any element information and their decoding is completely predicted by the previous I macroblocks and motion vectors. However, sometimes the I macroblock and motion vector cannot fully recover the jump macroblock before encoding, which will cause the compression distortion of the video. Based on this, this paper proposes the concept of the number of jump macroblocks as another characteristic parameter to evaluate the compression impairment. The larger the number of jump macroblocks, the higher the compression rate, but the more serious the distortion, while the smaller the number of jump macroblocks, the more the pixel information in the encoded video, and the better the decoded video quality.

### 3.2. Transmission Impairment Feature Extraction

Since it is difficult to obtain the network information of each node in the transmission process at the terminal in practical applications, this paper proposes two air-domain impairment characteristic parameters: strain impairment and block effect impairment and three time-domain impairment characteristic parameters: initial buffer duration, motion jump frequency, and motion jump average duration; thus, the video quality can be evaluated.

#### 3.2.1. Stretching Degree *D*_*s*_

Stretching refers to the distortion generated by the boundary of adjacent strips after decoding. The minimum object of this parameter is the strip of the video frame image, not the macroblock. Striping is a concept in video coding and decoding. A frame image usually has multiple strips and many macroblocks in a strip, and the purpose of setting strips is to prevent excessive error transmission during decoding and prediction. Therefore, the strain between strips is usually reflected on the edges in the horizontal direction, because strips are usually lined up horizontally side by side.

Assuming that strips *S*_*i*_, *S*_*i*−1_, and *S*_*i*+1_ are adjacent to each other up and down, *I*_*i*_(*n*, *m*) represents the brightness value of the pixel where the strip *S*_*i*_ is located at (*n*, *m*). Then, the degree of strain is expressed as

(4) $$\begin{array}{c} D_{s}=\left|\sum_{n=0}^{N-1}I_{i}\left(0,n\right)-\sum_{n=0}^{N-1}I_{i-1}\left(N-1,n\right)\right|+\left|\sum_{n=0}^{N-1}I_{i+1}\left(0,n\right)-\sum_{n=0}^{N-1}I_{i}\left(N-1,n\right)\right|. \end{array}$$

When calculating the overall strain effect of a frame, it is sufficient to average the degree of strain of the individual strips; i.e.,

(5) $$\begin{array}{c} D_{s,\text{frame}}=\frac{1}{n}\sum_{1}^{n}D_{s,n}. \end{array}$$

#### 3.2.2. Block Effect Damage *D*_*B*_

The degree of strain is for strips, while block effect damage is for macroblocks. The traditional block effect calculation method tends to count the block effect degree of all macroblocks and then average it into one frame. However, this approach is usually only applicable to a single image, and, for video, there are multiple frames per second, so the calculation will consume a lot of time. Therefore, this paper detects the possible damaged macroblocks and finally calculates the block effect degree of a frame by the possible damaged macroblock area.

#### 3.2.3. Block Effect Set

For two frames with the same average block effect level, if the damaged macroblocks are more concentrated in one frame, the quality of this frame is poorer. Therefore, the greater quality damage caused by multiple adjacent macroblocks with block effect is called “block effect set” in this paper. In this paper, we determine the quality of the whole frame according to the most serious block effect areas in a frame and cluster the block effect macroblocks to evaluate the combined block effect degree of each cluster.

#### 3.2.4. Time-Domain Impairment

When users watch videos, they often prefer to watch videos with poor clarity and to ensure the continuity of video playback. Therefore, the video is particularly important for the assessment of motion jump impairment. For motion jump impairment, whether it is frame repetition or frame freezing or initial buffering, the user feels the video lag. Therefore, in order to evaluate the time-domain impairment from the pixel domain, this paper proposes an algorithm to detect video jams. First, the pixel luminance difference between two adjacent frames is calculated to indicate the motion of the image sequence.

(6) $$\begin{array}{c} M=\frac{1}{w\times h}\left|I_{i}-I_{i-1}\right|, \end{array}$$

where *I*_*i*_ denotes the luminance signal of the first *i* frame and *w* and *h* denote the width and height of the image frame, respectively. The calculation result *M* reflects the motion of the image sequence, and a larger value indicates a more intense motion; a smaller value indicates a less significant difference between frames. When the value is less than a threshold *m*, it can be assumed that a motion jump may have occurred here. However, the repetition of the view may not be perceived by the human eye. Therefore, the algorithm requires that the value of *M* must be less than the threshold *m* for *n* consecutive frames and the best result is obtained when the value *m* is 0.3, which is *n* taken as follows. *N* is the total number of frames in the video sequence and *T* is the length of the video sequence:

(7) $$\begin{array}{c} n=2\times \frac{N}{T}. \end{array}$$

Based on the above formula, it has been possible to determine the occurrence of video playback jams. Considering the subjective perceptual characteristics of human eyes, the time-domain impairment is subdivided into three characteristic parameters for the time-domain impairment, which are initial playback delay, motion jump frequency, and average motion jump duration. These three parameters can be updated by real-time statistics each time the network lag is discerned.

## 4. BPNN-Based Video Quality Evaluation

### 4.1. Video Quality Evaluation Model Scheme for Sparring Sports

Combining the feature parameters proposed in Chapter 3, a BPNN-based video quality evaluation system model for sparring sports is proposed, and the system structure block diagram is shown in Figure 1.

Firstly, the video received by users is read in real time and then decoded by H.264 decoder. Here, the JM decoder is chosen, which is from the official source code of H.264 and has good support features. The quantization parameters, the number of jump macroblocks, and the frame sequence can be obtained directly from the decoder.

From the frame sequence, the strain parameter, block effect parameter, and aggregated block effect degree can be extracted by the formula in Chapter 3. Meanwhile, according to the motion jump detection algorithm proposed in Chapter 3, the occurrence of each motion jump can be detected from the frame sequence, and the duration of each occurrence and the position in the video where it occurs can be counted, so that the three parameters of initial buffering delay, jamming frequency, and average duration of jamming can be calculated.

After all the input parameters of the BPNN are obtained through data processing, the video quality scores in the training set are then trained to derive the weights of each neuron in the neural network. In this way, the predicted video quality scores can be obtained by extracting the above nine feature parameters from the video, processing them, and inputting them into the trained BPNN during testing and application.

### 4.2. BPNN Algorithm

The basic idea of BPNN is the gradient descent method, which uses the gradient search technique to minimize the mean squared error between the actual output value and the desired output value of the network. A typical three-layer BPNN is shown in Figure 2, with a topology consisting of an input layer, a hidden layer, and an output layer. For each neuron, the sigmoid function and gradient descent are usually utilized to predict the coefficients.

The basic BPNN algorithm consists of two processes: forward propagation of the signal and backward propagation of the error. That is, the error output is calculated in the direction from the input to the output, while the adjustment of the weights and thresholds is performed from the output to the input. In forward propagation, the input signal acts on the output node through the implied layer, and, after nonlinear transformation, the output signal is generated, and if the actual output does not match the desired output, it is transferred to the backward propagation process of the error. Backpropagation is to pass the output error back to the input layer through the hidden layer, apportion the error to all units of each layer, and use the error signal obtained from each layer as the basis for adjusting the weight of each unit. By adjusting the connection strength of the input nodes to the hidden layer nodes and the connection strength of the hidden layer nodes to the output nodes and the threshold value, the error decreases in the gradient direction, and, after repeated learning and training, the network parameters (weights and thresholds) corresponding to the minimum error are determined and the training is stopped. At this point, the trained neural network is able to process the input information of similar samples and output the information with the smallest error after nonlinear transformation by itself.

The important parameters and description of the learning process are presented as follows, based on the three-layer BPNN block diagram in Figure 2:

(1) Let the input parameters *X*_*i*_(*i*=1,2,…, *n*) denote the input features of the training set samples.
(2) Let the output parameters *Z*_*i*_(*i*=1,2,…, *L*) denote the prediction results obtained after the eigenvalues of the training set samples are passed through BPNN.
(3) Let the standard output *O*_*i*_(*i*=1,2,…, *L*) denote the standard result of the training set samples.
(4) Let the weight matrix *W* denote the coefficient matrix between the input layer output and the hidden layer input and the weight matrix *V* denote the coefficient matrix between the hidden layer output and the output layer input. As the model output obtained from each training set sample is compared with the standard output for learning, these two matrices are corrected by the gradient descent method. The matrices are corrected once for each sample until the input of the next sample, and finally the learning process of the network model meets the requirements.
(5) *g*(*x*) is the transfer function between the input and output of the hidden layer, and *f*(*x*) is the transfer function between the input and output of the output layer. Since the input features have been processed by the feature engineering related methods before the input layer, the input of the input layer is often equal to the output of the input layer. And, for BPNN, *g*(*x*) and *f*(*x*) can use the same sigmoid function, as shown in
  (8) $$\begin{array}{c} f\left(x\right)=g\left(x\right)=\frac{1}{1+e^{-x}}. \end{array}$$
(6) Set *a*_*i*_(*i*=1,2,…, *m*) as the hidden layer threshold, which is used to correct the input of the hidden layer; set *b*_*i*_(*i*=1,2,…, *m*) as the output layer threshold, which is used to correct the input of the output layer.
(7) Let *S*_*i*_(*i*=1,2,…, *m*) be the input of the hidden layer and *R*_*i*_(*i*=1,2,…, *p*) the input of the output layer. The number of nodes in the input layer is equal to the number of input features, which is set as *n* (in the model in this paper, *n* takes the number of features of the video 7), the number of nodes in the hidden layer is set as *m*, and the number of nodes in the output layer is set as *L* (in this model, only the video quality score is predicted, so *L* is taken as 1). The total number of input samples in the training set is *P*(*P*=1,2,…, *P*); *X*_*pi*_ is the *i* input component of the *p* sample. *W*_*ik*_ denotes the transfer weight from the first *i* node in the input layer to the first *k* node in the hidden layer. *V*_*kj*_ denotes the transfer weight from the first *k* node of the hidden layer to the first *j* node of the output layer.

Let the *p* sample input be the following:

(9) $$\begin{array}{c} X^{p}=\left(x_{p1},x_{p2},\ldots ,x_{pn}\right). \end{array}$$

Then, the input of the hidden layer is

(10) $$\begin{array}{c} S_{pj}=\sum_{i=1}^{n}x_{pi}\cdot w_{ij}-a_{i},\;j=1,2,\ldots ,m. \end{array}$$

The matrix form is written as

(11) $$\begin{array}{c} S^{p}=X_{1\times n}^{p}W_{n\times m}. \end{array}$$

The output of the hidden layer is

(12) $$\begin{array}{c} y_{pj}=g\left(s_{pj}\right)=g\left(\sum_{i=1}^{n}x_{pj}\cdot w_{ij}-a_{i}\right),\;j=1,2,\ldots ,m. \end{array}$$

Output layer input is

(13) $$\begin{array}{c} r_{pj}=\sum_{i=1}^{n}y_{pj}\cdot v_{ij}-b_{j},\;j=1,2,\ldots ,L. \end{array}$$

The output layer output is

(14) $$\begin{array}{c} z_{pj}=f\left(r_{pj}\right)=f\left(\sum_{i=1}^{n}y_{pi},v_{ij}-b_{j}\right),\;j=1,2,\ldots ,L. \end{array}$$

For all *P* samples, there is a global mean square error function that represents the measure of deviation of the sample as a whole between the sample output *Z*_*p*_ and the standard output *O*_*p*_ for each sample. The mean squared error function is denoted by *E*:

(15) $$\begin{array}{c} E=\frac{1}{2}\sum_{p=1}^{p}E_{p}=\frac{1}{2}\sum_{p=1}^{p}\sum_{t=1}^{L}{\left(e_{py}\right)}^{2}=\frac{1}{2}\sum_{p=1}^{P}\sum_{t=1}^{L}{\left(o_{pt}-Z_{pt}\right)}^{2}, \end{array}$$

where *E*_*p*_ denotes the first *p* sample error and *O*_*pt*_ is the *t* expected output of the *p* sample.

According to the derivation of gradient descent method, the output layer weight adjustment formula is

(16) $$\begin{array}{c} \Delta w_{jk}=-\eta \frac{\partial E}{\partial V_{jk}}=\eta \sum_{p=1}^{p}\left(O_{pj}-z_{pj}\right)\cdot z_{pj}\left(1-z_{pj}\right)\cdot y_{pj}, \end{array}$$

where *η* represents the learning efficiency and generally takes a value between [0, 1]. If the value of *η* is larger, the convergence speed increases, but it may lead to oscillation or even divergence; if the value of *η* is smaller, the training can converge steadily, but the learning speed is slower *η*.

Based on the derivation of gradient descent method, the implied layer weight adjustment formula is

(17) $$\begin{array}{c} \Delta w_{ki}=-\eta \frac{\partial E}{\partial w_{ki}}=\eta \sum_{p=1}^{p}\left(\sum_{j=1}^{m}\delta_{pj}v_{jk}\right)\cdot y_{pj}\left(1-y_{pj}\right)\cdot x_{pi}. \end{array}$$

Among them,

(18) $$\begin{array}{c} \delta_{pj}=\left(0_{pj}-z_{pj}\right)\cdot z_{pj}\left(1-z_{pj}\right). \end{array}$$

In summary, video quality evaluation using BPNN is divided into two main parts. The first part inputs the relevant feature parameters of the video to get a set of outputs (evaluated video quality scores) and then compares this set of outputs with the desired outputs (subjective quality scores) to derive the errors. The second part uses the gradient descent method to correct the two weight matrices *W* and *V*. After the two matrices are corrected, one iteration ends. This step is followed by the next sample input, and the correction of the weight matrices continues. Continuing in this order, the objective quality score of the output gradually approximates the subjective quality score and finally reaches the desired error accuracy, which represents the end of the BPNN learning process. With this trained BPNN model, the quality score of the video can be obtained from the feature parameters of the video, which is an objective assessment of the video quality.

## 5. Experimental Results and Analysis

### 5.1. Video Training Dataset and Subjective Evaluation

When people make subjective evaluations, they are able to give good or bad video image quality without the original video as a reference, even if most of the video images have never been seen before, based on their own a priori knowledge. This is mainly because people have seen videos of various qualities before. For neural networks, the prerequisite for supervised learning is the need for a priori knowledge of video quality, i.e., the need for a subjective quality assessment value of the video. In this paper, there are 24 original HD reference videos in the experimental database, which are from various sports topics on YouTube, including sports interviews, boxing commercials, and sports news. Each original video in the database corresponds to 180 distorted video sequences, which are recorded by terminals under different network conditions and contain real network transmission impairments, mainly varying degrees of airspace impairments and time-domain “lag.” In addition, the distortion videos also contain compression distortion for each compression parameter. The video set was given 3280 quality scores by 54 evaluators, and the video quality of the 320 video sequences was obtained by combining these quality scores, with the final quality score ranging from 1 to 100 indicating the worst to the best, with one decimal place for minimum precision. All evaluators watched the videos using the web page and scored them immediately after viewing.

### 5.2. Experimental Results and Analysis

The parameters of the final training neural network are as follows: the number of hidden layer nodes is 47, the momentum term is 0.95, and the initial value of the learning rate is 0.001, but it can be adjusted dynamically during the training process, the slope factor of the sigmoid function is −4.5, and the final minimum error is 0.0006. The test sample and the training set are one to four. The fitting diagram of subjective evaluation results and objective evaluation results of training samples and test samples has been given. As shown in Figures 3 and 4, the fitting scores reached 98.47% and 92.04%, respectively. According to the test results of the test materials, the correlation between the subjective evaluation results and the objective evaluation results is 92.04%, which has achieved an ideal effect.

Among them, the iterative training was stopped on the training set when the fit reached 98.47%, which indicates that there is a strong correlation between the selected feature parameters and the subjective quality scores and also avoids the overfitting of the training. The fit of the test set is 92.04%, which indicates that the quality evaluation results of this model are closer to the subjective quality scores.

In addition, the Standard Error (RE), Pearson's Correlation Coefficient (PCC), and Deviation Rate (DR) between the objective and subjective evaluation results of the proposed method are calculated and compared with Pulse Coupled Neural Network (PCNN), nonsubsampled shear wave transform (NSSWT), and orthogonal matching pursuit (OMP) methods, proving that the method in this paper has better performance in terms of accuracy and stability and the results are shown in Figures 5–7.

In this paper, we analyze the comparison for the missing feature parameter changes and the comparison for the added feature parameter changes, as shown in Figures 8 and 9. In Figure 8, missing any feature parameter, the final predicted fit decreases to different degrees, thus proving that the nine feature parameters are necessary. Meanwhile, it can be concluded from the graphical analysis that the quantization parameters, blurriness, average duration of jams, and frequency of jams have a greater impact on the video quality, which also compounds the daily concerns about the video quality. And, as shown in Figure 9, the quality prediction results are rather bad after adding parameters such as block flatness and bit rate, and the prediction results are somewhat enhanced after adding the location where the jams occur, but the extraction of this feature parameter will greatly increase the time complexity of the algorithm, and the result enhancement is not obvious, so this feature parameter is also discarded. In addition, this paper also tried to increase the real-time performance of the algorithm by extracting region of interest (ROI) and finally found that the real-time performance was not significantly enhanced, while the accuracy of quality assessment had a significant decline.

In this paper, we also try other regression algorithms such as Linear Regression (LR), Gradient Boosting Regression (GBR), and Support Vector Machine (SVM) regression models. The comparison of the fitting results of each regression algorithm is shown in Figure 10.

It can be seen that, among these four regression algorithms, the accuracy of BP neural network is the best. The effect of SVM and neural network is very close, and after several times of debugging the parameters of the objective function and kernel function, there is a slight difference between the optimal case and the result of neural network, so this paper finally uses BP neural network algorithm to fit the features to derive the video quality score.

## 6. Summary and Outlook

In this paper, we discuss the background and significance of video quality evaluation according to the development status of video and introduce the development status and trend of video quality evaluation methods. This paper analyzes in detail the compression damage and transmission damage suffered by the video and proposes nine parameters: quantization parameters, blurring degree, number of jumping macroblocks, strain degree, block effect, aggregated block effect degree, initial buffering time, average playback pause time, and playback pause frequency. Combining the proposed nine characteristic parameters affecting the video, this paper proposes a video quality evaluation system architecture. This architecture uses a BP neural network algorithm to fit the feature parameters, which can eventually output the predicted video quality scores. Finally, the proposed video quality evaluation method is experimentally simulated by the implemented system in this paper, and the accuracy of this paper is improved by 14.28% compared to the comparison algorithm.

The research work on video quality evaluation in this paper is only a small part in this field. At the same time, the research on video quality evaluation in this paper may have many areas for improvement and can be used as a direction for future research. The video quality evaluation method proposed in this paper is based on compression impairment and transmission impairment. However, in the actual network service system, the video quality may be affected by many subjective factors such as user terminal, user viewing environment, and user's subjective expectation for video. Therefore, a future research direction of this paper is to evaluate the video quality based on compression impairment and transmission impairment. Therefore, one of the future research directions of this paper is to quantitatively evaluate the subjective characteristics of users and add them to the objective video quality evaluation model in this paper, so that the evaluation of videos can be more accurate and more relevant to users.

## Figures and Tables

**Figure 1:** Network video quality evaluation system model.

**Figure 2:** Three-layer BPNN model.

**Figure 3:** The subjective evaluation value and objective evaluation value of training set.

**Figure 4:** The subjective evaluation value and objective evaluation value of training set.

**Figure 5:** BNPP compared with other video quality evaluation algorithms in terms of RE value.

**Figure 6:** BNPP compared with other video quality evaluation algorithms in terms of PCC value.

**Figure 7:** BNPP compared with other video quality evaluation algorithms in terms of DR value.

**Figure 8:** Effect of missing parameter features on prediction results.

**Figure 9:** Effect of adding parameter features on prediction results.

**Figure 10:** The comparison of accuracy of regression algorithms.

## Data Availability

The data used to support the findings of this study are available from the corresponding author upon request.
